The article "Recognition Method of Vehicle Cluster Situation Based on Set Pair Logic considering Driver's Cognition" was published in 2021. Journal: Comput Intell Neurosci.

# Recognition Method of Vehicle Cluster Situation Based on Set Pair Logic considering Driver's Cognition

**DOI:** 10.1155/2021/9809279

**Published:** 2021-09-04

**Authors:** Shijie Liu, Xiaoyuan Wang, Chenglin Bai, Huili Shi, Yang Zhang, Fusheng Zhong, Yaqi Liu

**Affiliations:** ^1^College of Electromechanical Engineering, Qingdao University of Science & Technology, Qingdao 266000, China; ^2^School of Transportation and Vehicle Engineering, Shandong University of Technology, Zibo 255000, China; ^3^Collaborative Innovation Center for Intelligent Green Manufacturing Technology and Equipment of Shandong Province, Qingdao 266000, China; ^4^School of Physics Science and Information Technology, Liaocheng University, Liaocheng 252000, China

## Abstract

The recognition of vehicle cluster situations is one of the critical technologies of advanced driving, such as intelligent driving and automated driving. The accurate recognition of vehicle cluster situations is helpful for behavior decision-making safe and efficient. In order to accurately and objectively identify the vehicle cluster situation, a vehicle cluster situation model is proposed based on the interval number of set pair logic. The proposed model can express the traffic environment's knowledge considering each vehicle's characteristics, grouping relationships, and traffic flow characteristics in the target vehicle's interest region. A recognition method of vehicle cluster situation is designed to infer the traffic environment and driving conditions based on the connection number of set pair logic. In the proposed model, the uncertainty of the driver's cognition is fully considered. In the recognition method, the relative uncertainty and relative certainty of driver's cognition, traffic information, and vehicle cluster situation are fully considered. The verification results show that the proposed recognition method of vehicle cluster situations can realize accurate and objective recognition. The proposed anthropomorphic recognition method could provide a basis for vehicle autonomous behavior decision-making.

## 1. Introduction

The road traffic system is a complex open system, integrating the human-vehicle-environment and other subsystems with high randomness, indeterminacy, and real-time capability. In recent years, with the rapid development of the transportation industry, the vehicle population has increased rapidly. The contradiction between humans, vehicles, and the environment has become more prominent. It is no longer possible to solve the contradiction between traffic supply and demand through road construction and expansion and conventional traffic control. With the development of new technologies such as the Internet of Things and Artificial Intelligence, advanced driving technologies such as intelligent driving and automated driving have become effective ways to alleviate the contradiction between supply and demand in traffic.

Vehicle cluster situation is the dynamic arrangement state and situation, which is automatically formed by the target vehicle and surrounding vehicles to complete their driving tasks. The vehicle cluster situation is formed and transferred under the human-vehicle-environment joint action and the traffic situation's core content [1]. Vehicle cluster situation is the link between the environment perception and driving behavior decision-making. Moreover, it is the comprehensive process result of traffic environment information and the basis for driving behavior decision-making. The research on vehicle cluster situations is helpful to analyze driving behavior and road traffic system in-depth and provides the theoretical basis for the research of intelligent driving and automated driving.

At present, many scholars have studied the analysis and modeling of the environment outside the vehicle. Guindel et al. [2] proposed a vision-based method with a deep convolutional neural network to detect the location of objectives and their orientations in traffic scenes. This method could robustly detect dynamic agents in road traffic environments to recognize traffic situations using onboard vision systems. Meyer-Delius et al. [3, 4] defined traffic situation as a series of meaningful states, using Hidden Markov Model to describe each traffic situation's probability distribution. The proposed model can simulate and identify traffic situations and predict the location of the tracked vehicle. They also proposed a traffic situation generalized learning model, which learns dynamic traffic situation characteristics and identifies situations. Käfer et al. [5] researched the recognition and prediction of the traffic situation at the intersection containing two vehicles. The vehicle movement database was used to estimate the trajectories of two vehicles 2–4 s in advance. The possible trajectories of the two vehicles constitute the possible traffic situation. Based on the vehicle's mutual visibility and the assumption of the driver's attempt to avoid the collision, an interactive model was established to identify and predict the traffic situation. Fu et al. [6] researched the behavior analysis method of distant vehicles using 3D Lidar, built upon convolution optimization and interacting multiple models framework. The proposed method could explore the traffic situation by estimating trajectory variation, analyzing position information, and determining behavior events. Lan et al. [7] studied the influence of driving behavior on vehicle cluster situations under the Internet of Vehicles. And they also researched the influence of factors on vehicle network situation and vehicle cluster situation, such as route selection, signal lights, and the roadside unit. Cao et al. [8] studied the interpretation, classification, and reasoning model of microscopic traffic situations using the case-based reasoning method. The proposed reasoning model can improve the system's reasoning description, continuous interpretation, and real-time inference capabilities of the traffic situation. Jerath et al. [9] studied the size of vehicle groups in self-organization under the intelligent and connected environment. And a generalized Ising model based on statistical mechanics was proposed to simulate traffic flow at the microscale and predict vehicle group distribution. Wang et al. [10] proposed a probability method to estimate vehicle cluster formation and evolution, including the division and reconstitution of vehicle clusters. In this study, the state of single vehicles is estimated by the Bayesian estimation method, the speed and position proximity of single vehicles is evaluated by probabilistic collision conditions, and the vehicle cluster state is identified by the density-based clustering method.

Most research of vehicle cluster situations only considers physical characteristics such as vehicle trajectories, and few studies consider driver and traffic flow characteristics. Wu et al. [11] determined the traffic situation map by the dynamic traffic entities' position in the target vehicle's interest region and discussed the mutual conversion relationship between situations with finite state automata. Zhang et al. [12] studied the transformation mechanism of vehicle group relationship in a dynamic and complex three-lane environment and analyzed the vehicle group in which the target vehicle was driving in different lanes. The transformation mechanism of vehicle group relationships under a time-varying environment is explored by identifying and changing the law of vehicle group relationships. Saeedmanesh et al. [13] explored the spatiotemporal relation of congested links and the congestion propagation of the traffic clustering situation in urban traffic networks. A static clustering method was developed to achieve rapid calculation of traffic networks situation and estimation of congestion propagation. Wang et al. [14] studied the reverse reconstruction method of vehicle group situations in urban road networks based on driver-vehicle feature evolution. The Gamma distribution theory was used to identify the vehicle group situation when the target vehicle arrived at the end of the study area. Hu et al. [15] presented a probabilistic framework for predicting traffic situations, which could jointly predict continuous motions and duration for multiple interacting road participants under any driving scenarios. Considering the premise of privacy protection of the driver, Wang et al. [16] constructed the reverse deduction model of vehicle group situation with travel time using a dynamic Bayesian network, which could realize the recognition and deduction of vehicle group situation. Focusing on the collective scenario understanding in a multivehicle system, Cavaliere et al. [17] proposed a consensus-based approach to lead multiunmanned vehicles to find agreement on the observed situation and build a group situation-based description of the scenario.

Vehicle cluster situation, which is the basis of decision-making, is perceived and recognized by the driver. Intelligent and automated driving require the anthropomorphic perception of vehicle cluster situations to make safe and efficient behavior decisions. Logic is a discipline used to study human thinking forms and laws, objectively describing human cognition of things. Some scholars researched the vehicle cluster situation based on fuzzy logic. Based on fuzzy logic, Wang et al. [18] introduced the concept of “force” in physics to represent the influence of surrounding vehicles on the target vehicle to describe the vehicle cluster situation objectively. The influence of the surrounding vehicle on target vehicle behavior was described with the concept of force. Moreover, the transformation mechanism of vehicle cluster situations under the dynamic evolution of driver's propensity is also studied. The dual random variations of vehicle cluster situations and drivers' propensity were modeled to explore the transformation mechanism. Fuzzy logic only considers the extent to which a proposition is true or false when giving real value to propositions. It is hard to judge the truth or falseness of the proposition with great uncertainty in some cases. Set pair logic fully considers the uncertainty and dynamic variability of things. It is a form of reasoning that corresponds more to the objective reality and can depict human cognition more objectively, comprehensively, and systematically. Set pair logic is applied in many fields [19–23].

Furthermore, the development of a study on the vehicle cluster situation based on set pair logic has multiple meanings. On the one hand, this research is one of the most critical contents of Connected and Automated Vehicles, which is closely related to driving safety. The vehicle cluster situation model and anthropomorphic recognition method based on set pair logic can fully express the certainty and uncertainty of the vehicle cluster situation, realize the accurate recognition of vehicle cluster situation, and represent traffic environment knowledge and driving conditions objectively. The recognition results are the anthropomorphic perception and cognition of traffic environment and driving conditions, providing the basic conditions for the autonomous behavior of Connected and Automated Vehicles. On the other hand, this research is also an essential part of human-machine-environment cooperation and interaction. The model based on set pair logic can take the factors of driver-vehicle-environment into overall consideration to provide the basis for the vehicle's decision-making. In a word, this research can provide an essential theoretical basis for developing the Connected and Automated Vehicle and conducting in-depth research of human-machine-environment interaction. In other words, this study has specific theoretical significance and application prospects.

From the literature review and the above analysis, it is easy to find that the research on vehicle cluster situations is the current research hotspot with certain theoretical significance and application prospects. So, it is necessary to study the recognition of vehicle cluster situations for the further development of Connected and Automated Vehicles. In view of this, the vehicle cluster situation model and recognition method are constructed by set pair logic based on our team's existing research to realize the anthropomorphic perception and cognition of traffic environment and driving conditions.

## 2. Set Pair Logic

### 2.1. Basic Concept

Set pair logic is a mathematical tool to deal with fuzzy and uncertain knowledge, depicting human cognition objectively. It can effectively analyze and process various uncertain information such as inaccurate, inconsistent, and incomplete information, explore the hidden knowledge, and reveal the potential law [24]. Pair principle refers to the existence of things in pairs: universal relation and unity of opposites. When a set is used to represent either side of a pair of things, the pair of things constitute a pair consisting of two sets, which is a set pair. The phenomenon of set pair is universal, and it is necessary to study mathematics and system on the basis of set pair, construct vehicle cluster situation model, and design recognition method of vehicle cluster situation.

According to the uncertainty principle, it is known that some system parameters cannot be determined when analyzing the microscopic level of the system. For human cognition, micro and macro are relative concepts. There is inevitable uncertainty when the macro- and microlevels of things are combined for overall consideration. The uncertainty comes from the relativity of hierarchy division, the fuzziness of hierarchical boundaries, and the dynamic migration and mutual conversion of system levels. Therefore, uncertainty must exist in the process and result from a problem's systematic study. The uncertain principle is also a derivation of the pair principle: the certainty and uncertainty of systems exist in pairs.

The pair principle and uncertainty principle are the two basic principles on which the set pair logic is based. In the study of vehicle cluster situations, the microscopic characteristics (such as vehicle features) and macroscopic characteristics (such as traffic density) should be comprehensively considered with the uncertainty of information. Therefore, the set pair logic is exceptionally suitable for vehicle cluster situation modeling and recognition.

Both fuzzy logic and set pair logic are methods used to describe human cognition of things logically. At the beginning of logic research, formal logic was built based on the classical set to study the certainty of laws of thinking, and the concept of two-valued logic was proposed. In two-valued logic, a proposition can only take two values, true or false. In contrast, a proposition can have multiple true values actually, which is multivalued logic. Three-valued logic is a particular multivalued logic expressing probability; that is, a proposition can take three values: true, false, or possible. In this regard, researchers study fuzzy thinking, language, and laws by using fuzzy mathematics such as the fuzzy set and membership functions, that is, fuzzy logic. Fuzzy logic could describe human cognition of things better by taking the extent to which a proposition is true or false as the true value. Fuzzy logic considers the fuzziness of the driver's cognition, but in some cases, it is hard to judge whether a proposition is true or false and the extent to true, with great uncertainty. For uncertainty, set pair logic is developed based on two-valued logic and fuzzy logic, which fully considers things' uncertainty and dynamic variability. Fuzzy logic separates “positive-indefinite-negative”, while set pair logic unites “positive-indefinite-negative”. Compared with fuzzy logic, set pair logic can depict human cognition and description of uncertain issues more objectively, comprehensively, and systematically.

### 2.2. Connection Number

The connection number is the set pair's characteristic function, reflecting research objects' different relationships and structures. It is also a structure-function with constructive and a certain form. The most basic connection number is the binary connection number, and its expression is

(1) $$\begin{array}{c} U=A+Bi, \end{array}$$

where *A* and *B* are nonnegative real numbers, which are certain and uncertain connection components, respectively; *i* ∈ [−1,1] is the value coefficient of uncertain connection component *B*. Let *N*=*A*+*B*, *a*=*A*/*N*, *b*=*B*/*N*, and *μ*=*U*/*N*; equation (1) can be transformed into

(2) $$\begin{array}{c} \mu =a+bi, \end{array}$$

where *a*+*b*=1. Equations (1) and (2) are collectively referred to as the binary connection number, connection number for short.

In binary connection number, *A*(*a*) is relatively certain, and *B*(*b*) is relatively uncertain, so that it can be called “certainty-uncertainty connection number”. Binary connection number can also be called “identical and different connection number”; in the research process, there is a relationship of “identical” and “same” between the set to be studied and the baseline set; *A*(*a*) and *B*(*b*) can be called the identical and different components, respectively. The form of a binary connection number is the same as a complex number, so it can also be called a complex connection number. However, the meaning of the binary connection number is different from a complex number. The basic operations of connection numbers include addition, numerical multiplication, multiplication, and vector operation.

Let *U*_1_=*A*_1_+*B*_1_*i* and *U*_2_=*A*_2_+*B*_2_*i* be two connection numbers; the addition operation is

(3) $$\begin{array}{c} U=U_{1}+U_{2}=\left(A_{1}+A_{2}\right)+\left(B_{1}+B_{2}\right)i. \end{array}$$

When *n*(*n* ≥ 3) connection numbers add up, there is

(4) $$\begin{array}{c} U=\overset{n}{\underset{j=1}{\sum }}U_{j}=\overset{n}{\underset{j=1}{\sum }}A_{j}+\overset{n}{\underset{j=1}{\sum }}B_{j}i. \end{array}$$

The connection numbers' addition meets commutative law and associative law. Let *α* be a real number; the numerical multiplication operation of connection number is

(5) $$\begin{array}{c} \alpha U=\alpha A+\alpha Bi. \end{array}$$

The product of two connection numbers is

(6) $$\begin{array}{c} U=U_{1}\cdot U_{2}=\left(A_{1}+B_{1}i\right)\left(A_{2}+B_{2}i\right)=A_{1}A_{2}+\left(A_{1}B_{2}+A_{2}B_{1}\right)i+B_{1}B_{2}i^{2}. \end{array}$$

It can be found that the product of two connection numbers is the quadratic function of *i*. Note that when *i* is only used as a marker, it is agreed that *i*^2^=*i*, since *i* is the representative of uncertain.

The connection number equation describes the state of the system, covering certain and uncertain components. A plane rectangular coordinate system is constructed with the *x*-axis as the certainty measure and the *y*-axis as the uncertainty measure. Then, the coordinate system is Determine-Undetermined Space, referred to as D-U Space or Set Pair Space (see Figure 1). The binary connection number determines the vector $\overset{⟶}{OM}$ in D-U Space, which is called the mapping of connection number *U* in the D-U Space. And the vector operation (expression of trigonometric function) of connection number is

(7) $$\begin{array}{c} U=r\left(\cos\theta +i\;\sin\theta \right), \end{array}$$

where *r* is the modulus of connection number, and *θ* is the argument of connection number, which can be calculated according to equations (8) and (9).

(8) $$\begin{array}{c} r=\sqrt{A^{2}+B^{2}}, \end{array}$$

(9) $$\begin{array}{c} \theta =\arctan\frac{A}{B}. \end{array}$$

### 2.3. Interval Number

Human perception and cognition of things is a “range” with uncertainty rather than an exact number, and the interval number is inherently uncertain. If *a* and *b* are real numbers, *a*, *b* ∈ *R* and *b* > *a*, then [*a*, *b*] is the interval number, where *a* is the lower bound of the interval number, and *b* is the upper bound. If the upper and lower bounds of the interval number are variables, they are usually marked as *x*^+^ and *x*^−^, and the interval number is marked as $\tilde{x}$, so the general form of interval number is

(10) $$\begin{array}{c} \tilde{x}=\left[x^{-},x^{+}\right], \end{array}$$

where *x*^−^, *x*^+^ ∈ *R* and *x*^+^ ≥ *x*^−^. The upper and lower bounds of the interval number define a one-dimensional interval. The length of the interval is *l*=*x*^+^ − *x*^−^. Interval numbers are a set of real numbers, and the variables of interval numbers ate uncertain components. The interval number is a set pair.

### 2.4. Transformation of Interval Number and Connection Number

For interval number $\tilde{x}=\left[x^{-},x^{+}\right]$, let

(11) $$\begin{array}{c} A=\frac{x^{-}+x^{+}}{2},\\ B=x^{+}-\frac{x^{-}+x^{+}}{2}. \end{array}$$

In combination with equation (1), the interval number can be transformed into a connection number, and the transformation equation of the interval number and the connection number is

(12) $$\begin{array}{c} U=\left(\frac{x^{-}+x^{+}}{2}\right)+\left(x^{+}-\frac{x^{-}+x^{+}}{2}\right)i,\;i\in \left[-1,1\right]. \end{array}$$

After the transformation from interval number into connection number, the expression of the trigonometric function of connection number can be gained according to equations (7)–(9).

(13) $$\begin{array}{c} U=r\left(\cos\theta +i\;\sin\theta \right),\\ r=\sqrt{{\bar{x}}^{2}+s_{x}^{2}},\\ \bar{x}=\frac{x^{-}+x^{+}}{2},\\ s_{x}=\frac{x^{+}-x^{-}}{2},\\ \theta =\arctan\frac{s_{x}}{\bar{x}}. \end{array}$$

## 3. Vehicle Cluster Situation Model and Recognition Method

### 3.1. Vehicle Cluster Situation Model

Vehicle cluster situation is the phase state, automatically formed by the driving state and relatively spatial-temporal relationship of the target vehicle and surrounding vehicles. The formation and transformation of the vehicle cluster situation are affected by various factors of the human-vehicle-environment. The vehicle cluster situation corresponds to the field of vehicle interaction. Three lanes are a typical complex scene of the urban expressway, so the following method will take three lanes as an example to introduce.

Driving behavior decisions should be made considering the macroindex, such as speed and density, and the microindex, such as the interaction between the surrounding vehicles. Therefore, considering the traffic flow characteristics, the interaction among vehicles can be abstracted as the interaction force based on the concept of “force” in physics. The resultant force exerted by each vehicle on the target vehicle is denoted as the force exerted by the lane on the target vehicle. The force exerted by the lane on the target vehicle could abstract the target vehicle's cluster situation. Suppose a vehicle exerts a positive influence on the target vehicle's selection of the lane where the vehicle is located. In that case, the vehicle exerts an attractive force on the target vehicle. Otherwise, it is a repulsive force. The effect size can describe the magnitude of the force. The effect size is mapped to an interval [−1,1] with the greatest attractive force represented by 1 and the greatest repulsive force represented by −1. According to equation (12), the interval number of force between vehicles can be transformed into a connection number. The modulus of the connection number of forces between vehicles can be calculated according to equations (8) and (13). Based on our team's existing research, the interval number, connection number, and the modulus of the connection number of the effect size are shown in Table 1. In the research, the modulus of the connection number of force between vehicles is distinguished into attractive force (positive number) with no sign and repulsive force (negative number) with a negative sign.

In the three-lane urban expressway (see Figure 2), the interest region is divided into 6 subregions according to the position of the target vehicle's front bumper. The subregions are left-front, left-rear, front, rear, right-front, and right-rear. The speeds of the target vehicle *n*_1_, left-front vehicle *n*_2_, left-rear vehicle *n*_3_, front vehicle *n*_4_, rear vehicle *n*_5_, right-front vehicle *n*_6_, and right-rear vehicle *n*_7_ are donated by *v*_*nj*_(*j*=1,2,…, 7). The relative distance between the target vehicle and the surrounding vehicles is donated by Δ*d*_2_, Δ*d*_3_, Δ*d*_4_, Δ*d*_5_, Δ*d*_6_, and Δ*d*_7_, respectively. The relative speed is marked as Δ*v*_2_≜*v*_*n*2_ − *v*_*n*1_, Δ*v*_3_≜*v*_*n*1_ − *v*_*n*3_, Δ*v*_4_≜*v*_*n*4_ − *v*_*n*1_, Δ*v*_5_≜*v*_*n*1_ − *v*_*n*5_, Δ*v*_6_≜*v*_*n*6_ − *v*_*n*1_, and Δ*v*_7_≜*v*_*n*1_ − *v*_*n*7_. The vehicle types are donated as *T*_*j*_∈ {small-sized vehicle, middle-sized vehicle, large-sized vehicle} (*j*=1,2,…, 7). The driving propensity of each driver is donated as *P*_*j*_ ∈ {Radical, Common, Conservative},  (*j*=1,2,…, 7).

Driving efficiency, driving safety, and driving comfort are the main factors for drivers to consider. Driving efficiency is mainly affected by average speed, while driving safety and driving comfort are mainly affected by traffic flow density. Hence, in addition to the traffic entity characteristics and vehicle group relationships mentioned above, such as vehicle type, driving propensity, relative distance, and relative speed, vehicle cluster situation should also cover the primary traffic flow macrocharacteristics, such as average speed and traffic flow density.

For the three parameters of traffic flow, there is a relationship of *q*=*k* · *v* among traffic volume *q*, speed *v*, and density *k*. In the actual study, the urban expressway's traffic flow state can be divided into three levels: smooth, slow, and congestion. The corresponding service levels of each traffic state are shown in Table 2.

The relative distance Δ*d*_*i*_ ∈ [0, +*∞*) between the target vehicle and the surrounding vehicle is divided into {danger, near, medium, far}. The relative speed Δ*v*_*i*_ ∈ (−*∞*, +*∞*) between the target vehicle and the surrounding vehicle is divided into {negative large, negative small, zero, positive small, positive large}. Considering the fuzziness and uncertainty of the driver's perception and cognition, the division of relative distance and relative speed are shown in Figures 3 and 4.

The boundary value [25] of the relative distance between “danger” and “near” is determined by

(14) $$\begin{array}{c} d_{1}=\frac{v_{n3}^{2}-v_{n1}^{2}}{2B_{\max}}+\tau v_{n3}+\lambda_{0}, \end{array}$$

where *τ* is the reaction time of the left-rear vehicle, *B*_max_ is the vehicle's maximum acceleration, and *λ*_0_ is the undetermined parameter. Equation (14) is the minimum distance to avoid collision between the target vehicle and the left-rear vehicle brake at the same acceleration when special events occur in front of the target vehicle. The boundary value of the relative distance between “near” and “far” is

(15) $$\begin{array}{c} d_{4}=D_{0}+\frac{{\left(v_{n3}-v_{n1}\right)}^{2}}{2acc}+\lambda_{1},\\ D_{0}=\frac{v_{n3}^{2}}{2B_{\max}}+\tau v_{n3}+\lambda_{2}, \end{array}$$

where *acc* is the acceleration of the target vehicle, and *λ*_1_ and *λ*_2_ are the undetermined parameters. *d*_2_ and *d*_3_ are the median of *d*_1_ and *d*_4_, respectively.

In order to ensure driving safety, the Time To Collision (TTC) can be used to evaluate the risk of collision. Taking the target vehicle and left-rear vehicle as an example, TTC can be calculated by

(16) $$\begin{array}{c} \text{TTC}=\left|\frac{\Delta d_{3}}{\Delta v_{3}}\right|. \end{array}$$

According to Minderhoud's statistics on driver's lane changing data and driver's subjective acceptable safety limit [26], the 5% quantile (2.6 s) and 25% quantile (5 s) of TTC were taken as the boundary value. It means that

(17) $$\begin{array}{c} v_{1}=-\frac{d_{1}}{2.6},\\ v_{2}=-\frac{d_{1}}{5}, \end{array}$$

where *v*_3_ and *v*_4_ are the opposite number of *v*_2_ and *v*_1_, respectively. Based on the data of section I-80 in NGSIM and empirical value, the boundary value of relative distance and relative speed are determined using cyclical training and the expert option method [27]. The boundary values are shown in Table 3.

### 3.2. Reduction of Vehicle Cluster Situation Model

There are 7^3^=343 kinds of vehicle cluster situations of the target vehicle, when the target vehicle is in the left, middle, and right lanes. The vehicle cluster situation is too complicated for the subsequent research, so it is necessary to reduce it.

First of all, the forces are only divided into attraction, zero, and repulsion, ignoring the magnitude. After this reduction step, the number of vehicle cluster situations of the target vehicle in the left, middle, and right lanes is 3^3^=27 for each one, a total of 81 vehicle cluster situations. When the target vehicle is in the left or right lane, it is hard for the target vehicle to perceive the separated lane's force directly. The force from the adjacent lane and the separated lane can be merged into the force of the side lane. The reduction rules are shown in Table 4. By this time, when the target vehicle is located in the middle lane, there are 3^3^=27 kinds of vehicle cluster situations; when the target vehicle is located in the left or right lane, there are 3^2^=9 kinds of vehicle cluster situations, respectively, for a total of 45 kinds.

When the force exerted by a lane on the target vehicle is zero, it is also a relatively good candidate lane.

Therefore, the force of zero is also regarded as an attractive force, and the force can be further reduced to attractive force and repulsive force. So there are 2^3^=8 kinds of vehicle cluster situations of the target vehicle located in the middle lane. There are 2^2^=4 kinds of vehicle cluster situations of the target vehicle located in the left and right lanes, respectively. After this step, the vehicle cluster situations were reduced to 16 kinds (see Figure 5).

### 3.3. Recognition Method of Vehicle Cluster Situation

During driving, the driver's perception of the traffic environment information is uncertain, and the driver gains uncertain information. The interval number can describe the certainty and uncertainty of the observed value objectively. Hence, the interval number can represent the driver's cognition and subjective judgment of the traffic environment information. However, there is no universally accepted method for comparing, sorting, and operating interval numbers [28]. To solve this problem, the interval number is transformed into the connection number based on the uncertainty system theory and the connection number of set pair logic [19]. Then, the recognition of the vehicle cluster situation is carried out. Therefore, the traffic environment information can be represented as the interval number, transformed into a connection number, and then transformed into the expression of the trigonometric function. Furthermore, the vehicle cluster situation recognition can be realized by the modulus of expression of the trigonometric function of the connection number.

The vehicle cluster situation is recognized based on the vehicle style of the target vehicle, vehicle style of surrounding vehicles, relative distance (considering the influence of driving propensity), relative speed (considering the influence of driving propensity), traffic flow density, and average speed. According to the 6 indexes, the force of each vehicle in the interest region on the target vehicle is recognized, and then the vehicle cluster situation of the target vehicle is determined. The recognition process of the vehicle cluster situation is shown in Figure 6. The procedure of the recognition of vehicle cluster situation is summarized in Algorithm 1.

### 3.4. Model Calibration

According to our existing research [27] and the division of each characteristic index (in the previous subsection), the interval numbers (7 forces on 6 indexes)were determined to obtain the interval number of reference characteristic values (see Table 5).

The driving propensity is mainly used to select the reference characteristic values of relative distance and relative speed. The vehicle type is mainly used to reduce the selection range of force without relying on the interval number. The interval numbers of reference characteristic values were transformed into connection numbers according to equation (12) (see Table 6). The moduli of connection numbers of reference characteristic values of vehicles' interaction force were calculated by equations (8) and (13) (see Table 7). At this point, the processing of the reference characteristic values of vehicles' interaction force was completed.

## 4. Results and Discussion

### 4.1. Example Application

Taking the target vehicle in the middle lane as an example, the traffic information of the target vehicle at a certain moment is given to recognize the vehicle cluster situation of the target vehicle. At this moment, the information acquired by the target vehicle is an exact value, which is a special connection number with an uncertain component of 0 (see Table 8, the numbers outside the bracket). Moreover, the moduli of the connection numbers of characteristic indexes of vehicles' interaction force to be recognized are calculated (see Table 8, the numbers inside the bracket).

According to Algorithm 1, the identical degree on the 6 characteristic indexes can be calculated. Taking the left-front vehicle as an example, the identical degrees between the force of left-front vehicle on a target vehicle and 7 kinds of forces on the relative distance are as follows:

(18) $$\begin{array}{c} a_{23}^{1}=\frac{52.3}{54}=0.9685,\\ a_{23}^{2}=\frac{44.7}{54}=0.8278,\\ a_{23}^{3}=\frac{48.1}{54}=0.8907,\\ a_{23}^{4}=\frac{44.1}{54}=0.8167,\\ a_{23}^{5}=\frac{39.7}{54}=0.7352,\\ a_{23}^{6}=\frac{38.2}{54}=0.7074,\\ a_{23}^{7}=\frac{36.9}{54}=0.6833. \end{array}$$

Among the identical degrees,

(19) $$\begin{array}{c} \underset{p=1,2,\ldots ,7}{\max}a_{23}^{p}=a_{23}^{1}=0.9685. \end{array}$$

Based on the principle of the greatest identical degree, the force of the left-front vehicle on the target vehicle shown in the relative distance is a strong attraction force. The identical degrees between the force of each vehicle in the interest region on the target vehicle and 7 kinds of forces on each characteristic index can be calculated to determine the type of force. Furthermore, the comprehensive force of each vehicle on the target vehicle is determined according to the moduli of forces' connection numbers (see Table 9).

Based on the driver's perception weight to different regions considering driving propensity, the comprehensive force of each lane on the target vehicle is calculated. And the vehicle cluster situation of the target vehicle is determined (see Table 10).

### 4.2. Verification of Recognition Method

In order to verify the reliability of the vehicle cluster situation model and recognition method, the confusion matrix, accuracy, precision, and recall were used to illustrate the performance of the model and recognition method. Accuracy, precision, and recall can be calculated by equations (20), (21), and (22), respectively.

(20) $$\begin{array}{c} \text{accuracy}=\frac{TP+TN}{TP+TN+FP+FN}, \end{array}$$

(21) $$\begin{array}{c} \text{precision}=\frac{TP}{TP+FP}, \end{array}$$

(22) $$\begin{array}{c} \text{recall}=\frac{TP}{TP+\text{FN}}, \end{array}$$

where *TP*, *TN*, *FP*, and *FN* are the sample sizes of true positive, true negative, false positive, and false negative, respectively.

In the verification process, the sample data is selected from the NGSIM dataset. In order to make sure of the labels of the sample data, 30 drivers (10 per driving propensity and 15 per gender) were selected to judge vehicle cluster situation. The 30 drivers recognized the vehicle cluster situations of all sample data to obtain the labels of sample data considering driving propensity. Only the sample data, which is uniformly recognized as the same vehicle cluster situation by all drivers with the same driving propensity, was selected as the verification dataset. In this process, 160 groups of data (10 for each kind of vehicle cluster situation) were extracted as the verification dataset.

The proposed method was validated by comparing it with the recognition method based on fuzzy logic and the driver's cognition results. The two models' recognition results were compared with drivers' cognition results to verify whether the models can objectively represent the driver's cognition of the vehicle cluster situation. The confusion matrixes of the comparison results are shown in Figure 7.

The results show that the overall accuracy of the recognition method of vehicle cluster situation based on fuzzy logic and set pair logic is 91.9% and 94.4%, respectively. For the different driving propensity, the accuracy of the method based on fuzzy logic is above 91%, and the accuracy of the method based on set pair logic is more than 93%. As for precision, the recognition method of vehicle cluster situation based on set pair logic is superior to the method based on fuzzy logic in most cases. Furthermore, the lowest precision of the recognition method based on set pair logic is higher than 81%. The results of the recall are similar to precision; that is, the recognition method based on set pair logic is better than the method based on fuzzy logic in most cases. Moreover, the lowest recall of the recognition method based on set pair logic is higher than 80%. Overall, the recognition method of vehicle cluster situation based on set pair logic has higher accuracy, precision, recall, and better performance. In other words, the recognition method of vehicle cluster situation based on set pair logic is better than the method based on fuzzy logic. The verification result of the recognition method of the vehicle cluster situation proposed in this research proves that the recognition result is more objective. According to the verification, we can further infer that this method is suitable for the anthropomorphic cognition of Connected and Automated Vehicles, and this method can provide a basis for anthropomorphic decision-making.

## 5. Conclusions

In this research, the certain and uncertain traffic environment information is fully explored using connection number and interval number methods. A new vehicle cluster situation model and recognition method are proposed based on the set pair logic theory considering the characteristics of human cognitive systems. The proposed model and method fully consider traffic entities' characteristics in the target vehicle's interest region, grouping relationships, and macroscopic traffic flow characteristics to objectively represent the target vehicle's vehicle cluster situation. The interval numbers of reference characteristic values are determined considering the driving propensity of the target vehicle driver. The interval number is converted into the connection number and then transformed into the expression of the trigonometric function. The transformation process acknowledges the certainty and uncertainty of the vehicle cluster situation. The certainty of vehicle cluster situation is reflected in the upper and lower bounds of interval number and the certain component of connection number. The uncertainty of the vehicle cluster situation is reflected in the fluctuation of upper and lower bounds of interval number and the uncertain component of connection number. The force is recognized according to the moduli's identical degree, which acknowledges the interaction between certainty and uncertainty (the moduli are calculated from the certain and uncertain component of the connection number). Based on the modulus of force and the influence of driving propensity on driver's cognition, the comprehensive forces from each vehicle and each lane on the target vehicle are determined to recognize the vehicle cluster situation further.

Compared with the existing research, the proposed recognition method of vehicle cluster situation is based on the comprehensive cognition of the driver. It is the practical application of human logic reference theory in the perception and cognition of the traffic environment. The proposed recognition method presents the relatively certain information and relatively uncertain information of origin data and the interaction information of two kinds of information. Certainty, uncertainty, and the interaction between the two are unique characteristics of the human cognitive system, which have not been considered by existing studies of vehicle cluster situations. The recognition result is theoretically more objective and reasonable from the method based on the characteristics of human cognition. Furthermore, it is more in line with the needs of a Connected and Automated Vehicle for anthropomorphic decision-making. Compared with the recognition method based on fuzzy logic, the performance of the recognition method based on set pair logic shows higher accuracy, precision, and recall as a whole. The verification results show that the vehicle cluster situation model and recognition method proposed in this study can objectively represent the road traffic conditions and achieve accurate recognition.

In general, the method proposed in this research can accurately and objectively recognize the vehicle cluster situation from the perspective of human cognition. This study could provide a basis for anthropomorphic intelligent decision-making of Connected and Automated Vehicles and promote the development of Connected and Automated Vehicles. In addition, the results can also further the research of human-vehicle-environment cooperation and interaction.

## Figures and Tables

**Figure 1:** Mapping of the connection number U in the D-U Space.

**Figure 2:** Vehicle cluster situation of the target vehicle in the basic section of the three-lane urban expressway.

**Figure 3:** Division of relative distance.

**Figure 4:** Division of relative speed.

**Figure 5:** Division of vehicle cluster situation.

**Figure 6:** Recognition process of vehicle cluster situation.

**Figure 7:** Confusion matrix of recognition results of vehicle cluster situation. (a) Recognition results of vehicle cluster situation based on set pair logic. (b) Recognition results of vehicle cluster situation based on fuzzy logic. The comparison results show that the recognition method based on set pair logic proposed in this research is better than the recognition method based on fuzzy logic as a whole. (The precision is in the gray square at the bottom, the recall is in the gray square at the right, and the accuracy is in the blue square at the bottom right corner. The results of the blue, orange, and red font colors are the model performance under the driving propensity of conservative, common, and radical, respectively. The results of the black font color are the overall performance.

**Algorithm 1:** Recognition of vehicle cluster situation.

**Table 1:** Set pair representation of force.

Force		Strong repulsion (SR)	Middle repulsion (MR)	Weak repulsion (WR)	Zero	Weak attraction (WA)	Middle attraction (MA)	Strong attraction (SA)
Effect size	Interval number	[−1, −0.7)	[−0.7, −0.3)	[−0.3, 0)	0	(0, 0.3]	(0.3, 0.7]	(0.7, 1]
	Connection number	−0.85 + 0.15i	−0.5 + 0.2i	−0.15 + 0.15i	0	0.15 + 0.15i	0.5 + 0.2i	0.85 + 0.15i
	Modulus of connection number	−0.86	−0.54	−0.21	0	0.21	0.54	0.86

**Table 2:** Service level of urban expressway basic section.

Service level	Density (pcu/km/lane)	Speed (km/h)	Maximum service traffic volume (pcu/h/lane)
Smooth	*k* ≤ 32 (small)	*v* ≥ 54.5 (large)	1600
Slow	32 < *k* ≤ 50 (medium)	40 ≤ *v* < 54.5 (medium)	2100
Congestion	*k* > 50 (large)	*v* < 40 (small)	2100

**Table 3:** Boundary value of relative distance and relative speed considering driving propensity.

Parameter	*d*_1_	*d*_2_	*d*_3_	*d*_4_	*v*_1_	*v*_2_	*v*_3_	*v*_4_
Radical	8.2	22.5	36.7	51.3	−3.3	−1.6	1.6	3.3
Common	12.6	25.8	40.1	60.5	−4.8	−2.5	2.5	4.8
Conservative	22.3	38.3	54.4	70.4	−8.4	−4.5	4.5	8.4

**Table 4:** Reduction rules of the force of the side lane.

The force from the adjacent lane	The force from the separated lane	The force exerted by the side lane on the target vehicle
Attractive force	Attractive force	Attractive force
Attractive force	Zero	Attractive force
Attractive force	Repulsive force	Zero
Zero	Attractive force	Attractive force
Zero	Zero	Zero
Zero	Repulsive force	Zero
Repulsive force	Attractive force	Repulsive force
Repulsive force	Zero	Repulsive force
Repulsive force	Repulsive force	Repulsive force

**Table 5:** Interval number of the reference characteristic values.

Force	Driving propensity	Target vehicle type	Surrounding vehicle type	Relative distance	Relative speed	Traffic flow density	Average speed
SA	Radical	Small or middle or large	Small or middle	[22.5, 70.5]	[1.4, 5.1]	[0, 51]	[34,75]
	Common			[25.8, 83.6]	[2.2, 7.2]		
	Conservative			[38.3, 91.8]	[3.7, 12.3]		

MA	Radical	Small or middle or large	Small or middle	[16.8, 60.9]	[1.2, 4.6]	[20, 54]	[25, 69]
	Common			[20.6, 72.1]	[1.8, 6.4]		
	Conservative			[31.9, 81.1]	[3.2, 11.2]		

WA	Radical	Small or middle or large	Small or middle or large	[11.2, 67.1]	[−0.1, 3.8]	[25, 55]	[29, 71]
	Common			[15.3, 79.4]	[−0.2, 5.5]		
	Conservative			[25.5, 87.8]	[−0.3, 9.4]		

Zero	Radical	Small or middle or large	Small or middle or large	[10.5, 61.5]	[−2.4, 3.5]	[24, 56]	[35, 68]
	Common			[14.8, 74.7]	[−3.6, 5.1]		
	Conservative			[24.7, 81.6]	[−6.5, 8.9]		

WR	Radical	Small or middle or large	Small or middle or large	[7.2, 55.7]	[−2.8, 3.4]	[26, 59]	[28, 61]
	Common			[11.1, 66.7]	[−4.1, 4.9]		
	Conservative			[19.6, 75.6]	[−7.1, 8.6]		

MR	Radical	Small or middle or large	Middle or large	[3.6, 53.9]	[−3.4, 3.3]	[28, 64]	[25, 58]
	Common			[5.5, 64.2]	[−4.7, 4.8]		
	Conservative			[9.8, 73.2]	[−8.6, 8.4]		

SR	Radical	Small or middle or large	Middle or large	[0, 52.2]	[−6.6, 1.6]	[31, 100]	[22, 52]
	Common			[0, 61.7]	[−6.8, 2.5]		
	Conservative			[0, 71.3]	[−11.7, 4.5]		

**Table 6:** Connection number of the reference characteristic values.

Force	Driving propensity	Target vehicle type	Surrounding vehicle type	Relative distance	Relative speed	Traffic flow density	Average speed
SA	Radical	Small or middle or large	Small or middle	46.5 + 24*i*	3.25 + 1.85*i*	25.5 + 25.5*i*	54.5 + 20.5*i*
	Common			54.7 + 28.9*i*	4.7 + 2.5*i*		
	Conservative			65.05 + 26.75*i*	8 + 4.3*i*		

MA	Radical	Small or middle or large	Small or middle	38.85 + 22.05*i*	2.9 + 1.7*i*	37 + 17*i*	47 + 22*i*
	Common			46.35 + 25.75*i*	4.1 + 2.3*i*		
	Conservative			56.5 + 24.6*i*	7.2 + 4*i*		

WA	Radical	Small or middle or large	Small or middle or large	39.15 + 27.95*i*	1.85 + 1.95*i*	40 + 15*i*	50 + 21*i*
	Common			47.35 + 32.05*i*	2.65 + 2.85*i*		
	Conservative			56.65 + 31.15*i*	4.55 + 4.85*i*		

Zero	Radical	Small or middle or large	Small or middle or large	36 + 25.5*i*	0.55 + 2.95*i*	40 + 16*i*	51.5 + 16.5*i*
	Common			44.75 + 29.95*i*	0.75 + 4.35*i*		
	Conservative			53.15 + 28.45*i*	1.2 + 7.7*i*		

WR	Radical	Small or middle or large	Small or middle or large	31.45 + 24.25*i*	0.3 + 3.1*i*	42.5 + 16.5*i*	44.5 + 16.5*i*
	Common			38.9 + 27.8*i*	0.4 + 4.5*i*		
	Conservative			47.6 + 28*i*	0.75 + 7.85*i*		

MR	Radical	Small or middle or large	Middle or large	28.75 + 25.15*i*	−0.05 + 3.35*i*	46 + 18*i*	41.5 + 16.5*i*
	Common			34.85 + 29.35*i*	0.05 + 4.75*i*		
	Conservative			41.5 + 31.7*i*	−0.1 + 8.5*i*		

SR	Radical	Small or middle or large	Middle or large	26.1 + 26.1*i*	−2.5 + 4.1*i*	55.5 + 24.5*i*	37 + 15*i*
	Common			30.85 + 30.85*i*	−2.15 + 4.65*i*		
	Conservative			35.65 + 35.65*i*	−3.6 + 8.1*i*		

**Table 7:** Moduli of connection numbers of reference characteristic values.

Force	Driving propensity	Target vehicle type	Surrounding vehicle type	Relative distance	Relative speed	Traffic flow density	Average speed
SA	Radical	Small or middle or large	Small or middle	52.3	3.7	36.1	58.2
	Common			61.9	5.3		
	Conservative			70.3	9.1		

MA	Radical	Small or middle or large	Small or middle	44.7	3.4	40.7	51.9
	Common			53	4.7		
	Conservative			61.6	8.2		

WA	Radical	Small or middle or large	Small or middle or large	48.1	2.7	42.7	54.2
	Common			57.2	3.9		
	Conservative			64.6	6.7		

Zero	Radical	Small or middle or large	Small or middle or large	44.1	3	43.1	54.1
	Common			53.8	4.4		
	Conservative			60.3	7.8		

WR	Radical	Small or middle or large	Small or middle or large	39.7	3.1	45.6	47.5
	Common			47.8	4.5		
	Conservative			55.2	7.9		

MR	Radical	Small or middle or large	Middle or large	38.2	3.4	49.4	44.7
	Common			45.6	4.8		
	Conservative			52.2	8.5		

SR	Radical	Small or middle or large	Middle or large	36.9	4.8	60.7	39.9
	Common			43.6	5.1		
	Conservative			50.4	8.9		

**Table 8:** Connection numbers and moduli of characteristic indexes of vehicles' interaction force to be recognized (connection number is outside the bracket, and modulus is inside the bracket).

Surrounding vehicle	Driving propensity	Target vehicle type	Surrounding vehicle type	Relative distance	Relative speed	Traffic flow density	Average speed
Left-front vehicle	Radical	Small	Small	54 (54)	4.2 (4.2)	21 (21)	52 (52)
Left-rear vehicle			Small	42 (42)	2.9 (2.9)	21 (21)	52 (52)
Front vehicle			Small	43 (43)	1.2 (1.2)	45 (45)	47 (47)
Rear vehicle			Middle	28 (28)	−0.2 (0.2)	45 (45)	47 (47)
Right-front vehicle			Middle	52 (52)	2.4 (2.4)	42 (42)	46 (46)
Right-rear vehicle			Large	23 (23)	0.7 (0.7)	42 (42)	46 (46)

**Table 9:** Recognition results of the force of each vehicle on the target vehicle.

Surrounding vehicle	Driving propensity	Target vehicle type	Surrounding vehicle type	Relative distance	Relative speed	Traffic flow density	Average speed	Force of vehicle
Left-front vehicle	Radical	All forces	SA ∼ WR	SA	SA	SA	MA	SA
Left-rear vehicle			SA ∼ WR	Zero	Zero	SA	MA	WA
Front vehicle			SA ∼ WR	Zero	WA	WR	WR	WR
Rear vehicle			All forces	SA	WA	WR	WR	WR
Right-front vehicle			All forces	SA	WA	WA	MR	WA
Right-rear vehicle			WA ∼ SR	SA	WA	WA	MR	WR

**Table 10:** Recognition result of vehicle cluster situation of the target vehicle.

Lane of target vehicle	Lane	Comprehensive force	Vehicle cluster situation
Middle lane	Left lane	Attraction (MA)	*T*_6_
	Middle lane	Repulsion (WR)	
	Right lane	Repulsion (WR)	

## Data Availability

The data used to support the findings of this study are available from the corresponding author upon request.
